# Noninvasive Method for Predicting the Expression of Ki67 and Prognosis in Non-Small-Cell Lung Cancer Patients: Radiomics

**DOI:** 10.1155/2022/7761589

**Published:** 2022-03-16

**Authors:** Wei Yao, Yifeng Liao, Xiapeng Li, Feng Zhang, Haifeng Zhang, Baoli Hu, Xiaolong Wang, Li Li, Mei Xiao

**Affiliations:** ^1^Department of Oncology, The Fifth Affiliated Hospital of Sun Yat-sen University, Zhuhai 519000, China; ^2^Department of Cardiothoracic Surgery, Huaihe Hospital of Henan University, Kaifeng, China

## Abstract

**Purpose:**

In this study, we aimed to develop and validate a noninvasive method based on radiomics to evaluate the expression of Ki67 and prognosis of patients with non-small-cell lung cancer (NSCLC). *Patients and Methods*. A total of 120 patients with NSCLC were enrolled in this retrospective study. All patients were randomly assigned to a training dataset (*n* = 85) and test dataset (*n* = 35). According to the preprocessed F-FDG PET/CT image of each patient, a total of 384 radiomics features were extracted from the segmentation of regions of interest (ROIs). The Spearman correlation test and least absolute shrinkage and selection operator (LASSO), after normalization on the features matrix, were applied to reduce the dimensionality of the features. Furthermore, multivariable logistic regression analysis was used to propose a model for predicting Ki67. The survival curve was used to explore the prognostic significance of radiomics features.

**Results:**

A total of 62 Ki67 positive patients and 58 Ki67 negative patients formed the training set and test training dataset and test dataset. Radiomics signatures showed good performance in predicting the expression of Ki67 with AUCs of 0.86 (training dataset) and 0.85 (test dataset). Validation and calibration showed that the radiomics had a strong predictive power in patients with NSCLC survival, which was significantly close to the effect of Ki67 expression on the survival of patients with NSCLC.

**Conclusion:**

Radiomics signatures based on preoperative F-FDG PET/CT could distinguish the expression of Ki67, which also had a strong predictive performance for the survival outcome.

## 1. Introduction

Lung cancer is one of the leading malignant tumours worldwide with a high incidence rate and high mortality. Non-small-cell lung cancer (NSCLC) is the most common pathological type of lung cancer in all pathological types, accounting for 85% of all lung cancer patients [1, 2]. Because of the lack of early specific clinical symptoms, lymph node metastasis or distant metastasis has often occurred before diagnosis, which has a major impact on the treatment and prognosis. The five-year survival rate of lung cancer is less than 20% [3], although with the emergence of new drugs or treatment methods to improve the survival rate of lung cancer patients, at the same time, the same treatment method in time, the patients reflect a huge difference. Therefore, new biomarkers related to patient outcomes are needed to stratify the prognostic risk of patients.

Ki-67 is a nuclear protein expressed in the active phase of the cell cycle, except the G0 phase. The proliferation index (PI) of Ki-67 has been widely used as a marker of cell proliferation. Previous studies have shown high Ki-67 expression negative effect on disease-free survival, relapse-free survival, and overall survival in non-small-cell lung cancer [4–6]. The expression level of Ki-67 still has many challenges in clinical practice. In addition, these invasive methods are not only invasive but also may lead to bleeding, pneumothorax, and increase the possibility of tumour metastasis. Imaging technology can directly or indirectly reflect histopathological changes caused by the expression of genes and cytokines. Radiomics features can be used to quantify the spatial distribution of image pixels and grayscale and to reflect the corresponding molecular pathological changes at the microscopic level [7].

Radiomics is a new method of medical imaging research, which is a new noninvasive technology using medical imaging analysis and data in-depth analysis. The workflow of radiomics includes (1) medical image preprocessing, (2) ROI segmentation, (3) radiomics feature extraction, and (4) feature dimension reduction model establishment. Lots of clinical endpoints are associated with radiomics, in lung cancer, including survival time [8], differentiation of benign and malignant pulmonary nodules [9–11], and recurrence and distant metastasis [12, 13]. In recent years, the use of radiomics to decode tumour genotypes has attracted more and more attention. One study [14] has shown that the prediction model combined with radiomics characteristics and clinical risk factors may promote the individualized prediction of PD-L1 expression in patients with NSCLC. At the same time, many studies have explored the use of radiology to determine the EGFR mutation status in lung cancer tissues [15–19].

In the face of patients with NSCLC, targeted personalized treatment of precision medicine has gradually become the guiding ideology of treatment. The spatiotemporal heterogeneity of tumours limits the reuse of invasive biopsy in tumour patients [20]. Medical imaging determines tumour heterogeneity, which means that it is an ideal way to capture tumour heterogeneity through noninvasive means. Therefore, radiomics can be used as a potential molecular substitute to optimize the treatment selection and management of cancer [21]. To judge the expression of Ki67 in patients with NSCLC by noninvasive and easily available radiomics is of positive significance for the prognosis stratification of patients with NSCLC.

## 2. Methods

### 2.1. Patients

This study was reviewed and approved by the ethics committee of our unit, and according to the ethical principles, the relevant informed consent of the audience was exempted. We retrospectively collected the records of 316 patients from January 2010 to February 2016. After screening, 120 eligible patients were finally included in the study. The inclusion criteria were as follows: (a) confirmed NSCLC by postoperative pathology, (b) undergoing 18F-FDG PET/CT scanning within 2 weeks before any impaired operation, and (c) underwent surgery or other standard radiotherapy and chemotherapy, according to the treatment guidelines. The exclusion criteria were as follows: (a) partial loss of images, (b) received radiotherapy, chemotherapy, or other treatments for the tumour before the scan, (c) confirmed other types of cancer before the scan, (d) tumours too small to delineate or FDG negative uptake, and (e) no postoperative pathological reports. We randomly divided the patients into a training dataset (*n* = 84) and test dataset (*n* = 36), with a ratio of 7 : 3. Patients' characteristics with NSCLC are shown in Table 1. The Ki-67 index was reported in pathological reports, and its principle was calculated by the percentage of positive cells. The low expression of Ki-67 was defined as a positive staining of ≤40%, and the high expression of Ki-67 was more than 40% [22]. Information about survival time in this study was obtained through the patient's normative review or telephone.

### 2.2. Image Acquisition

Patients underwent PET/CT imaging using 18F-FDG, with a purity >99%, which came from GE minitrace II, Tracelab FDG preparation (GE Healthcare, Milwaukee, Wisconsin). All PET/CT scans were performed in a free-breathing mode, but no action was taken to correct the motion. Patients need to fast for more than 6 hours before the examination, and their blood glucose should be controlled below 7 mmol/L. Patients were intravenously injected with 18F-FDG (4 MBq/kg) and underwent a PET/CT scan of the skull base to the upper part of the thigh. A three-dimensional pet model was used. The matrix was 192 × 192, and the exposure time was 2 min/bed. Low-dose spiral CT was performed at 120–140 kV. After CT attenuation correction, time-of-flight, and point spread function algorithms were used to reconstruct PET images, including two iterations and 24 subsets.

### 2.3. Radiomics Processing Flow

PyRadiomics (https://pypi.org/project/pyradiomics/), an open-source tool, was used to process images and extract imaging features. Image biomarker Standardization Initiative (IBSI) guidelines [23] were considered to be the key guiding spirit of this work. We have preprocessed the image, which ensures the consistency of the three axial scales of the image in three dimensions. A total of 384 radiomics features were extracted from preprocessed PET/CT images, including first-order and higher-order features, which contained shape, histogram, gray-level dependency matrix (GLDM), gray-level co-occurrence matrix (GLCM), gray-level size zone matrix (GLSZM), and gray-level run length matrix (GLRLM). All features were processed by standard score normalization, which was undoubtedly to ensure normalization of data. Because the dimension of feature space is high, we compared the similarity of each feature pair. If the Pearson Correlation Coefficient (PCC) value of the feature pair was larger than 0.90, one of them was removed. After the process of relevance selection, the dimension of the feature space was reduced, and each feature was independent of the others. Then, we used the LASSO method to further select features, which is characterized by fitting the generalized linear model, variable selection, and complexity adjustment at the same time (Figure 1). The standardization steps of LASSO include determining the optimized hyperparameter *λ*, ensuring the minimum deviation of the model. Features that were with nonzero coefficients were preserved for the model. Multiple parameters with meaningful coefficients were used to form the final R-score.

### 2.4. Statistical Analysis

R software (version 4.0.4, https://www.Rproject.org) and SPSS statistical software (version 21.0; IBM) were used for statistical analysis in our study. We first compared the clinical information of the training set and the test set randomly and ensured that the two groups were not interfered with by other factors. All statistical tests were two-sided, with a significance level of 0.05. The PPC and LASSO were used for feature selection. Receiver operating characteristic (ROC) analysis was used to test the diagnostic performance of the radiomics model. We used the decision curve analysis (DCA) curve to judge the difference between R-score and other clinical features. We used the survival curve to judge the stratification ability of Ki67 and R-score on the prognosis of patients with NSCLC.

## 3. Results

### 3.1. Clinical Characteristics of Patients

We divided the patients with NSCLC (74 men, 46 women) into two groups, including the training dataset (*n* = 85) and the test dataset (*n* = 35). The clinical characteristics of the patients are summarized in Table 1. In these two groups, we found that there was no clear statistical difference in the clinical characteristics between the training dataset and the test dataset (*P* > 0.05).

### 3.2. Selection and Establishment of a Radiomics Model

By PCC and LASSO, a total of six important radiomic features were selected (Figure 2). We established a formula, using selected radiomic features, for predicting the expression of Ki67 in patients with NSCLC:

(1) $$\begin{array}{c} R-\text{score}=0.722*\text{HaralickCorrelation}\_\text{angle }45\_\text{offset }7+0.023*\text{Correlation}\_\text{AllDirection}\_\text{offset }1\_S\;D+0.339*GLCM\text{Entropy}\_\text{AllDirection}\_\text{offset }1\_S\;D\\ +0.35*\text{Inertia}\_\text{angle }45\_\text{offset }7-0.181*\text{ShortRunEmphasis}\_\text{angle }90\_\text{offset }1+0.08*\text{Maximum }3\;D\text{ Diameter}+0.168. \end{array}$$

Through training dataset and test dataset, R-score showed good resolution (Figure 3). In the training dataset, the area under curve (AUC) was 0.86 (95% CI, 0.78–0.94) and accuracy was 0.82 (95% CI, 0.73–0.90) with sensitivity 0.85 and specificity 0.79. In the test dataset, the AUC was 0.85 (95% CI, 0.71–0.98) and accuracy was 0.83 (95% CI, 0.66–0.93) with sensitivity 0.94 and specificity 0.72. To further test our model, we drew calibration curves on two datasets, and the results showed that R-score was accurate and generalized in predicting the expression of Ki67 (Figure 4).

### 3.3. The Prognosis of Patients with NSCLC

Follow-up data were collected from October 2010 to January 2021. The mean and median follow-up periods were 58.35 (95% CI, 52.89–63.81) and 56.50 (range, 8.00–110.00) months, respectively. We found that the positive expression of Ki67 could be a good prognostic factor (Figure 5). Then, we used R-score to group the patients, which also achieved great prediction results (Figure 6).

### 3.4. DCA for R-Score and Other Factors

To better explore the role of radiomics in patients with NSCLC, we used the DCA method for analysis. We defined size as the product of the tumour's long diameter and short diameter. In lobulation, speculation, shape, and boundary pleural, if there is no or no abnormality, we count it as 1; otherwise, it was 2. We defined Cscore as the sum of the abovementioned four indicators. Through the DCA curve, we could conclude that the omics model has better application ability (Figure 7).

## 4. Discussion

In previous studies, it was difficult to achieve great Ki67 prediction results using CT or enhanced CT alone [24, 25]. We used PET data, which can well add tumour metabolic information and achieve better classification. In this study, we used PET/CT radiomics features to investigate the expression of Ki67 and the prognosis of patients with NSCLC. Through the image before treatment, we obtained a radiomics signature to predict the expression of Ki67 and defined its prognostic significance, including Maximum3DDiameter, GLCMEntropy, Inertia, HaralickCorrelation, Correlation, and ShortRunEmphasis. At the same time, we also verified that radiomics just like Ki67 has guiding significance for prognosis in patients with NSCLC. A total of 384 radiomics features were extracted from the segmentation of ROIs in PET/CT. To remove redundant data and achieve better classification results, we used PCC and LASSO methods commonly used in feature selection [26, 27]. Maximum3DDiameter is an important indicator of tumour size. This index was included in the model, so in DCA comparison, we compared the model with tumour size (product of long diameter and short diameter) and determined a better predictive value. A gray-level co-occurrence matrix (GLCM) is a histogram of co-occurring grayscale values at a given offset over an image, and GLCMEntropy is an important index to reflect the degree of confusion of a two-dimensional gray-level co-occurrence matrix, which has been reflected in previous studies [28]. In head and neck cancers, inertia features [29] showed a correlation with epidermal growth factor receptor (EGFR). At the same time, it is related to the expression of Ki67 in lung cancer tissues in our research, suggesting that this texture parameter may be related to tumour heterogeneity and prognosis. Haralick texture features could contain information about image texture features, such as quality, grayscale linear correlation, contrast, the number and nature of existing boundaries, and the complexity of the image, which has been studied to explore its relationship with tumour mutation [30] and recurrence [31]. ShortRunEmphasis is often applied in the impact radiomics model. Shang-Wen Chen [32] showed that the feature extracted from PET/CT is related to the mutation of carcinogenesis in colorectal cancer. Through these key features, our model shows good predictive power (two datasets' AUCs more than 0.8).

In the previous studies [8, 27, 33], radiomics showed a great ability to predict survival. However, the interpretability and rationality of the model have been questioned [34]. Therefore, we used radiomics to predict Ki67 and further explained its role in prognosis. As seen in Figures 5 and 6, radiomics shows a hierarchical predictive ability of clinical outcomes similar to Ki67. Since it has been confirmed that Ki67 is an independent predictor of lung cancer [6, 35], the predictive ability of the radiomics model for survival of lung cancer patients can be largely explained.

Our research has some limitations. First of all, this is a retrospective study of a small dataset without external validation, which may introduce selection bias. Secondly, we only studied the expression of Ki67 in the prognosis of patients with lung cancer and did not consider the influence of other genes. Further research is necessary for the comprehensive evaluation of other genes.

## 5. Conclusions

Radiomics characteristics based on 18F-FDG PET/CT can distinguish the expression of Ki67, and it also has a strong ability to predict survival. This technical method will not only increase the patient's additional financial pressure or physical harm but also can achieve precise management of patients with NSCLC.

## Figures and Tables

**Figure 1:** Least absolute shrinkage and selection operator for selecting features.

**Figure 2:** Selected features and coefficients.

**Figure 3:** Receiver operating characteristic curve in the training dataset and test dataset.

**Figure 4:** The calibration curve in the training dataset and test dataset.

**Figure 5:** The Kaplan–Meier curve of Ki67.

**Figure 6:** The Kaplan–Meier curve of *R*-score.

**Figure 7:** The decision curve analysis.

**Table 1:** Clinical characteristics of patients.

Clinical features	Total	Training dataset	Test dataset
No. of patients	120	85	35
Mean age (95% CI)	55.58 (53.19–57.98)	55.46 (52.63–58.29)	55.87 (51.18–60.59)
*Sex*			
Male	74 (62%)	51 (60%)	23 (66%)
Female	46 (38%)	34 (40%)	12 (34%)
*TNM stage*			
I	39 (33%)	25 (29%)	14 (40%)
II	60 (50%)	46 (54%)	14 (40%)
III	21 (17%)	14 (17%)	7 (20%)
*Lobulation*			
Yes	84 (70%)	62 (73%)	22 (63%)
No	36 (30%)	23 (27%)	13 (37%)
*Spiculation*			
With	61 (51%)	40 (47%)	21 (60%)
Without	59 (49%)	45 (53%)	14 (40%)
*Shape*			
Irregular	59 (49%)	38 (45%)	21 (60%)
Regular	61 (51%)	47 (55%)	14 (40%)
*Boundary pleural*			
Invasion	75 (63%)	52 (61%)	23 (66%)
Noninvasion	45 (37%)	33 (39%)	12 (34%)

## Data Availability

The data used to support this study are available from the corresponding author upon request.
